The article "Assessing the environmental performance of optimized commercial refrigerators with alternative refrigerants and remote monitoring system: A cradle-to-grave life cycle assessment" was published in 2024. Journal: Heliyon.

# Assessing the environmental performance of optimized commercial refrigerators with alternative refrigerants and remote monitoring system: A cradle-to-grave life cycle assessment

**DOI:** 10.1016/j.heliyon.2024.e29753

**Published:** 2024-04-18

**Authors:** Ramoon Barros Lovate Temporim, Alessia Di Giuseppe, Fabiana Frota de Albuquerque Landi, Andrea Nicolini

**Affiliations:** a CIRIAF - Interuniversity Research Center on Pollution and Environment "Mauro Felli", Via G. Duranti 67, 06125, Perugia, Italy; b Department of Engineering, University of Perugia, Perugia, Italy; c Norwegian Institute for Sustainability Research, NORSUS, Stadium 4, 1671, Kråkerøy, Norway

**Keywords:** Life cycle assessment, Refrigeration system, Refrigerants gases, Optimization systems

## Abstract

Refrigerators, as other cooling systems, are responsible for a significant parcel of anthropogenic emissions since they are essential and heavy appliances that use energy during its lifespan and are loaded with refrigerant gases. Three types of commercial refrigerators and their new versions, with incorporated CO2 as refrigerant gas and an wireless system for maintenance monitoring (WSMM) were investigated to evaluate how optimization could impact on the environmental performance during their entire life cycle. This study conducted a comprehensive Life Cycle Assessment (LCA) of the refrigerators, from the production to their end-of-life. The findings revealed that the use phase and the raw materials were responsible for most of the environmental impact throughout the refrigerators' life cycle. Key impact categories such as Fossil Resource Scarcity, Freshwater Eutrophication, and Global Warming were particularly affected, largely due to the electricity mix in the use phase. Additionally, the extraction and production of raw materials, specifically steel and copper, made significant contributions to Terrestrial Ecotoxicity and Human Carcinogenic Toxicity categories. The optimization measures impacted mainly in the energy consumption during the use phase, resulting in a notable reduction of approximately 57 % for models that underwent refrigerant change and 60 % for the model that underwent both refrigerant change and electronic system installation. As a result of decreased energy consumption, there was a significant decrease of 13 %–16 % across all impact categories, underscoring the positive environmental implications of these optimization strategies.

## List of abbreviations

A: Model A
B: Model B
C: Model C
EU: European Union
FRS: Fossil Resource Scarcity
FEW: Freshwater Eutrophication
GWP: Global Warming Potential
HCT: Human Carcinogenic Toxicity
HFC: Hydrofluorocarbons
ISO: International Organization for Standardization
LCA: Life Cycle Assessment
OPT: Optimized
R452A: Blend of Pentafluoroethane(HFC R125), 2,3,3,3Tetrafluoroprop1ene – (HFO R1234yf), and Difluoromethane (HFC R32)
R490: Propane
R744: Carbon dioxide
TRE: Terrestrial Ecotoxicity
WEEE: Waste from Electrical and Electronic Equipment
WSMM: Electronic System for Maintenance Monitoring

The article "Assessing the environmental performance of optimized commercial refrigerators with alternative refrigerants and remote monitoring system: A cradle-to-grave life cycle assessment" was published in 2024. Journal: Heliyon.

## 1 Introduction

Refrigerators are essential appliances in both households and commercial establishments, offering a convenient and reliable solution for storing and preserving food, beverage and medicines. Currently, there are approximately 120 million active commercial refrigerators worldwide [1]. As living standards improve, the importance of maintaining a robust cold chain becomes increasingly evident. This critical chain plays a crucial role in preventing spoilage, extending the shelf life of products, and enhancing overall food safety [[2], [3], [4]]. By inhibiting the growth of bacteria and harmful pathogens, refrigeration effectively prevents foodborne illnesses, reducing the need for chemical additives in industrialized food production. The continuous advancements in freezing technologies have facilitated the rapid growth of new food markets, most notably the frozen food sector. Additionally, the evolving food landscape, with a growing reliance on prepared food options, has significantly influenced the lifestyle choices of urban populations, thereby increasing the demand for refrigeration appliances [5]. Furthermore, it is worth noting that the refrigeration manufacturing sector plays a substantial role in the global economy, providing employment opportunities for approximately 15 million people worldwide.

Countries such as the United States, Ireland, United Kingdon, Sweden, and Germany have an annual per capita consumption of frozen food reaching approximately 50 kg [5]. The global frozen food market, valued at 219.9 billion USD in 2018, is projected to experience substantial growth, estimated to increase by almost 30 % by 2023, reaching a value of USD 282.5 billion [6].

However, the refrigerator manufacturing industry has a substantial environmental footprint, encompassing the materials used in their production, the energy consumed during their use phase, and the potentially harmful refrigerants employed [7]. While numerous studies have explored the environmental impacts of cold chains, these investigations often focus on the entire chain, which includes factors such as agricultural food production, thereby overshadowing the specific impact of the cold chain responsible for food preservation [3,[8], [9], [10]]. Recent research has shed light on the significant contribution of refrigerator production and usage to overall environmental impacts.

The article "Assessing the environmental performance of optimized commercial refrigerators with alternative refrigerants and remote monitoring system: A cradle-to-grave life cycle assessment" was published in 2024. Journal: Heliyon.

This article is structure to outlines the current state of the refrigeration-based food preservation sector and its challenges related to environmental emissions. After identifying key issues in material usage, energy consumption, and end-of-life considerations, we propose an environmental impact analysis using the LCA methodology to quantify critical phases of the product life cycle and evaluates optimized versions of the analysed refrigerators. Following, in the Materials and Methods section, we introduce the LCA methodology and provide technical descriptions of each analysed refrigerator model and its optimized versions. The Results section presents inventory details for each model and the outcomes for the selected impact categories. In the Discussion section, we analyze results, compare with existing literature, suggest improvements in critical phases of the product life cycle, and conduct a comparative analysis between original and optimized refrigerator models.

### 1.1 Literature review

Refrigeration is an energy-intensive process with significant implications for the environment. As the cold production chains expand worldwide, the demand for energy continues to rise. Refrigeration is a major consumer of electricity, accounting for approximately 17 % of global electricity demand [11]. Studies have shown that refrigeration is responsible for more than 60 % of electricity usage in cold warehouses, contributing to about 70 % of greenhouse gas emissions in cold storage facilities [1,12]. In commercial establishments like supermarkets, the refrigeration system typically constitutes 30–60 % of total electricity consumption [1].

Ageing components in refrigerators can lead to increased energy waste, resulting in consumption levels that exceed the labelled values by 40–60 %. However, addressing this excessive consumption is possible through the repair of affected components and the adoption of predictable maintenance practices [7]. In fact, the constant advancement of refrigeration equipment is a significant concern that drives manufacturers, researchers, and policymakers to seek efficient and sustainable solutions [13].

In the study conducted by De Masi et al., 2023 [14], a LCA of two industrial refrigerators with different insulation technologies revealed that insulation has a minor impact on the environment. However, the transportation systems emerged as a substantial factor shaping the overall environmental footprint. This underscores the importance of addressing transportation efficiency in addition to insulation technologies to effectively minimise the environmental impact of refrigeration systems [14].

The article "Assessing the environmental performance of optimized commercial refrigerators with alternative refrigerants and remote monitoring system: A cradle-to-grave life cycle assessment" was published in 2024. Journal: Heliyon.

Refrigerant systems use refrigerants that can be harmful to the environment and Human Health due to their toxicity [1]. Extensive research has focused on finding substitute refrigerants that are as efficient as their predecessors but more environmentally friendly, in compliance with the Kyoto Protocols [15] and F-Gas regulations [16]. Alternative refrigerants such as R-290 (propane) and R-744 (carbon dioxide) have emerged as promising options. These alternatives offer lower environmental impact, reduced global warming potential, non-toxicity, and non-flammability. They can also be used in existing systems with minor modifications [17].

Growing awareness of the environmental impacts of the cold sector has prompted the development of international policies and initiatives focused on mitigating these effects. These efforts target greenhouse gas emissions, energy efficiency, and sustainable refrigeration practices, reflecting a global commitment to reducing the environmental footprint of cold chain and refrigeration systems. The Kigali Amendment to the Montreal Protocol [18] is particularly significant, as it aims to gradually reduce global production and consumption of hydrofluorocarbons (HFCs). Implementation of this amendment is crucial, as without it, HFC emissions from the refrigeration sector could reach 3–4 Gt CO_2_-eq by 2050 [19].

Previous research has conducted comparative assessments to explore the environmental consequences linked to diverse materials employed in the manufacturing of refrigerators. These studies have investigated energy consumption and greenhouse gas emissions specifically associated with two foamers: HFC-245fa (pentafluoropropane) and pentane, as documented by Johnson, 2004 [20]. Furthermore, McCulloch and Lindley, 2003 [21] performed a comprehensive life-cycle inventory analysis to evaluate the overall environmental impact of HFC-134a throughout the entire production process of refrigerators. Hwang examined the life-cycle climate performance of different refrigerants using collected data [22]. Campbell and McCulloch, 1998 [23] focused on assessing the greenhouse gas emissions linked to refrigerants during both their usage and disposal stages. It is important to note that these investigations primarily concentrated on examining the environmental impact of distinct materials utilized in refrigerators separately [7]. Consequently, there is a pressing need for comprehensive and integrated studies to thoroughly evaluate the environmental impact of refrigerators from a holistic perspective.

The electronic system for maintenance monitoring (WSMM) encompasses a network of interconnected physical devices, appliances, and objects capable of collecting and sharing data through embedded sensors and software. In the realm of refrigeration systems, WSMM technology can optimize performance, improve energy efficiency, and enhance food safety while minimizing waste. Real-time monitoring, predictive maintenance, and automated alerts facilitated by WSMM enable precise control of temperature and humidity levels, thereby promoting sustainability and cost-effectiveness in refrigeration systems [24]. Moreover, smart devices offer higher energy efficiency potential and generate significant data regarding their functionality and environmental conditions [5]. Manufacturers can analyze repair and maintenance requirements, explore usage-failure correlations, and effectively manage the product's life cycle, especially in terms of monitoring energy efficiency and component replacements within the WSMM-installed system [[25], [26], [27], [28]].

The article "Assessing the environmental performance of optimized commercial refrigerators with alternative refrigerants and remote monitoring system: A cradle-to-grave life cycle assessment" was published in 2024. Journal: Heliyon.

Finally, In Litardo et al., 2023 [29], a systematic review of peer-reviewed LCA articles on different active cooling or air conditioning systems was conducted, revealing that those utilising renewable energy sources generally exhibit lower life cycle impacts, in terms of GWP (Global Warming Potential), than their conventional counterparts [29].

## 2 Materials and Methods

The methodology employed in this study, spanning from the in situ data collection phase to the life cycle impact assessment and interpretation of results, is illustrated in Fig. 1.

**Fig. 1:** Methodology Implemented in the LCA study.

The data utilized in the present LCA study are derived from manufacturing company questionnaires and checklists. The collected data span each phase of the product life cycle, encompassing aspects such as raw material production, transportation of components, manufacturing, transportation of final products to customers, use phase, and end-of-life of refrigerator components.

Life Cycle Assessment (LCA) is a methodology that comprehensively evaluates the environmental impact of products and processes, considering all relevant environmental factors throughout their life cycle. By quantifying energy and material consumption, as well as waste generation, LCA enables the identification of opportunities to optimize and improve the environmental performance of products and processes. LCA follows the principles and requirements outlined in International Organization for Standardization (ISO) 14040:2006a [30] and 14044:2006b [31], which include goal and scope definition, life cycle inventory analysis, life cycle impact assessment, and interpretation. The LCA model was developed using SimaPro V9.4.0.2 [32], a commercial software designed for LCA modelling. The model was based on the Environmental Product Declaration - Household Refrigeration Appliances, specifically the PSR 2000:1 version, which is currently under revision [33].

The article "Assessing the environmental performance of optimized commercial refrigerators with alternative refrigerants and remote monitoring system: A cradle-to-grave life cycle assessment" was published in 2024. Journal: Heliyon.

### 2.1 Goal and scope

This paper presents a comprehensive and holistic approach which is essential for assessing the environmental sustainability of the cold chain, including the often-overlooked impacts of cold chain facilities themselves and the identification of effective interventions to mitigate these impacts. A cradle-to-grave LCA was conducted in this study, focusing on three types of commercial refrigerators and their optimized versions.

LCA methodology, a widely accepted approach in sustainability analysis, to comprehensively evaluate the environmental impact of refrigeration systems throughout their life cycle [7,28,34]. By applying LCA, the research aims to assess the environmental consequences of refrigerator usage, providing valuable insights into its overall environmental performance and identifying opportunities for sustainability improvement.

The LCA examined the environmental impact of refrigerant substitution and the implementation of WSMM technologies, aiming to understand and mitigate the environmental footprint of refrigerators. The findings provide valuable insights into the potential reduction of environmental impacts through these optimizations. This research serves as a powerful tool for manufacturers and consumers in making informed decisions regarding the environmental sustainability of refrigeration systems.

The objectives of this study were to assess the environmental impacts of three types of refrigerators, including the identification of significant impacts in terms of life cycle phases, materials, and processes. Additionally, the study sought to evaluate the environmental performance improvement achieved using alternative refrigerant gases and the implementation of electronic technologies that monitor the appliance performance during the use phase, i.e. WSMM. It aims to contribute to literature with primary data obtained from a large producer in central Italy.

#### 2.1.1 Declared unit

The declared unit correspond to a single unit of each refrigerator model and its respective optimized version. Additionally, according to other studies [13,35], a functional unit based on the refrigerated capacity of each model per year was proposed to enhance the comparison between the original and optimized models. This approach ensures a clear and concise assessment of the differences between the two models, original and optimized, particularly as the WSMM increases the refrigerator lifespan.

#### 2.1.2 System, time, and geographic boundaries

The system boundaries encompass the entire supply chains involved in refrigerator manufacturing, from the production of raw materials to the end-of-life stage of the refrigerator. The representation of these system boundaries can be observed in Fig. 2.

The article "Assessing the environmental performance of optimized commercial refrigerators with alternative refrigerants and remote monitoring system: A cradle-to-grave life cycle assessment" was published in 2024. Journal: Heliyon.

**Fig. 2:** System boundaries.

The data used in this analysis was collected within the European Union area. The raw materials were sourced from various countries, while the manufacturing plant is situated in central Italy. The time boundary for the assessment was set at a 10-year lifespan, comprising 7 years of standard use and an additional 3 years of extended use, as determined by the manufacturer and supported by other studies [[35], [36], [37]].

### 2.2 Refrigerators

Three different refrigerator models were examined, each designed to meet specific temperature requirements. Model A is a negative temperature refrigerator intended for frozen foods, Model B is a positive temperature refrigerator designed for refrigerated foods, and Model C is a negative temperature refrigerator specifically designed for ice cream storage. Detailed descriptions of these models and their corresponding optimization modifications can be found in Table 1. The products description is relevant for designing the use phase.

**Table 1:** Characteristics of Models A, B, and C and their optimized versions. Data obtained from a manufacturer in central Italy in 2021.

Standard Characteristics	Unit	Model A	Model B	Model C
Temperature of operation	°C	−18 to −15	−1 to +7	−16 to −10
Type of food	–	Frozen Food	Fresh Food	Ice Cream
Display area	m^3^	4.06	6.34	1.43
Weight	kg	649	640	510
Refrigerant		R290	R744	R452a
Defrost system		Hot Gas	Compressor Off	Reverse Cycle
Daily consume	kWh	38.50	18.42	40.32
Environmental conditions	°C/%RH	25/60	25/60	35/75
Dimensions	M	1.98 X 0.85 X 2.30	2.58 X 1.15 X 2.30	2.18 X 1.11 X 1.18
Capacity	liters	1432	1772	285
Power supply	V, ph, Hz	230/1/50	230/1/50	400/3/50
Average lifespan	years	7 + 3	7 + 3	7 + 3
**Optimized model**	**refrigerant**	**R744**	**R744**	**R290**
**Daily consume**	**kWh**	**33.50**	**15.52**	**34.50**

Table 1 lists all the technical characteristics of the models analysed in the first box. Subsequently, the optimizations carried out in terms of refrigerant replacement and quantities are reported.

#### 2.2.1 Data collection, data quality and life cycle inventory

The model was developed considering the following phases: raw material production, which includes all materials and processes involved in the production of refrigerator components; transportation of components; manufacturing, involving processes, energy demand for forming and assembling refrigerator components, emissions from processes, refrigerant losses, and waste management; transportation of final products to customers; use phase, focusing on electricity consumption; and end-of-life considerations, covering transportation, treatment, disposal, and recycling of refrigerator components.

The article "Assessing the environmental performance of optimized commercial refrigerators with alternative refrigerants and remote monitoring system: A cradle-to-grave life cycle assessment" was published in 2024. Journal: Heliyon.

The data collection process took place on-site during a comprehensive survey conducted at a manufacturing company located in Central Italy. The survey encompassed various aspects of both the manufacturing process and the product lifecycle. Raw material data was calculated based on the refrigerators' component inventory and substance leakage, while energy demands, including electricity from grid and photovoltaic sources, as well as natural gas, diesel, gasoline, and emissions from the manufacturing process, were directly measured on-site. For the use phase, energy consumption (electricity) was obtained from the supplier, considering the real operation of the refrigerators under different usage conditions and seasons. Transportation data for raw materials and final products was estimated by considering the distances between suppliers, the manufacturing plant, and the end consumers. The end-of-life scenario considered the degree of disassembly of the refrigerator's materials, with separable materials identified as recyclable and non-separable materials undergoing treatments such as burning or landfilling. The Design for Disassembly strategy was implemented to simplify the removal of specific electric and electronic components, helping recyclers comply with the Waste from Electrical and Electronic Equipment (WEEE) Directive [38]. Secondary data used for the modelling phase in SimaPro was sourced from the ecoinvent V3.8 database [39].

The optimization of the systems involved two main aspects: the adoption of new refrigerants and the implementation of WSMM sensing. Three different refrigerants were utilized: R290 (propane), R744 (CO2), and R452A (a blend of Pentafluoroethane - HFC R125, 2,3,3,3-Tetrafluoroprop-1-ene - HFO R1234yf, and Difluoromethane - HFC R32), considered alternative refrigerants [40]. The specific quantities for each refrigerator model are outlined in Table 1. The performance improvement of the system with the implementation of WSMM was evaluated as follows. By installing the WSMM system, it was estimated that efficiency could be enhanced through preventive maintenance, reducing the duration of inadequate refrigerator operation, which directly impacts power consumption. To estimate failures and damages occurring throughout the lifespan of the refrigerators, statistical records of system failures without the WSMM system were utilized. The monitored parameters included condenser fan damage, condenser dirt accumulation, evaporator fan damage, refrigerant gas loss, compressor malfunction, and high ambient temperature. The occurrence frequency and average detection time for each parameter were recorded. Based on this data, it was possible to determine the rate of compressor activation increase needed to compensate for the malfunctioning of other components, resulting in higher electricity consumption. Furthermore, the permanent compressor damage caused by excessive activation could be identified.

The article "Assessing the environmental performance of optimized commercial refrigerators with alternative refrigerants and remote monitoring system: A cradle-to-grave life cycle assessment" was published in 2024. Journal: Heliyon.

#### 2.2.2 Life cycle impact assessment

Initially, the ReCiPe Midpoint (H) V1.1 [41] method was used to evaluate which the 18 midpoint impact categories would be relevant. The method is based on commonly accepted policy principles and utilizes a timeframe of 100 years. Five of those environmental indicators were selected as focus of this evaluation: GWP [15], Fossil Resource Scarcity (FRS), Freshwater Eutrophication (FWE), Terrestrial Ecotoxicity (TRE), and Human Carcinogenic Toxicity (HCT).

Global Warming Potential is based on IPCC 2013 method measured in kg CO2 eq.is related to the concentration of greenhouse gases in the atmosphere. Notably these gases can cause a rise in the global average temperature and, consequently, the incidence extreme climate events and, the loss of fauna and flora balances. In this method, greenhouse gases are multiplied by a characterization factor reflecting their damage potential in global warming in comparison to CO_2_.

Additionally, the ReCiPe Endpoint (H/A) summarized results in three endpoint areas of protection, i.e., human health, ecosystems, and resources.

## 3 Results

### 3.1 Life cycle inventory

The refrigerator's inventory and their optimized versions are presented in Supplementary Materials - Table 1. The structure was designed based on the Product Category Rules PSR 2000:1. A simplification of the components was done by grouping similar materials into larger groups, such as cardboard, plastics, steel, wood, electronic components, and others. This approach follows the strategy adopted by Gasia et al., 2021 [34].

During the production phase, mass allocation was performed assigning the ratio of energy consumption needed to produce the refrigerators under investigation. Therefore, total consumption of fuels, grid and photovoltaic electricity, and heat reported by a traditional manufacturer in central Italy was divided by the whole factory production considering the mass of manufactured products. Emissions of atmospheric pollutants from industrial processes and the management of generated waste were also recorded. The transportation phase included the supply of raw materials to the production site and the distribution of finished products to global customers according to the manufacture data from 2021.

The article "Assessing the environmental performance of optimized commercial refrigerators with alternative refrigerants and remote monitoring system: A cradle-to-grave life cycle assessment" was published in 2024. Journal: Heliyon.

Throughout the product's lifespan, the energy consumption of each model was estimated. The optimized models considered an electricity consumption reduction attributed due to precise maintenance assigned by the electronic systems, i.e, WSMM. These models also contain alternative refrigerants than the traditional HFC-134a. Notably, the variations in components between the original and optimized models were minimal, with similar material quantities and a weight difference of less than 0.5 % of the total system weight. The weight of the WSMM sensing system was negligible compared to the overall system weight. At the end of the product's life, these materials were classified as recycled, incinerated, or buried based on the producer's disassembly levels.

### 3.2 Impact assessment results

#### 3.2.1 Midpoint level - normalisation

The process of normalising the results revealed five impact categories, which account for over 82 % of the total impact load of the analysed refrigerator models. The normalisation factors and detailed results of normalisation for all impact categories are shown in Supplementary Materials - Table 2, Table 3. Main results are presented in Table 2.

**Table 2:** Normalised ReCiPe (H) results.

Impact category	Model A		Model B		Model C	
	Standard	Optimized	Standard	Optimized	Standard	Optimized
HCT	64 %	66 %	70 %	71 %	59 %	61 %
FRS	7 %	7 %	5 %	5 %	8 %	8 %
FEW	5 %	4 %	3 %	3 %	5 %	5 %
TRE	5 %	5 %	6 %	6 %	5 %	5 %
GWP	3 %	3 %	2 %	2 %	4 %	4 %
Total	84 %	85 %	86 %	87 %	82 %	83 %

**Table 3:** Characterization of standard and optimized models and calculated variations.

CAT	Unit	A			B			C		
		St	Opt	Δ	St	Opt	Δ	St	Opt	Δ
*FRS*	*kg oil e.*	1.51E+04	1.32E+04	13 %	7.95E+03	6.86E+03	14 %	1.63E+04	1.38E+04	15 %
*FWE*	*kg P e.*	6.41E+00	5.61E+00	12 %	3.52E+00	3.06E+00	13 %	6.94E+00	5.91E+00	15 %
*GWP*	*kg CO2 e.*	5.64E+04	4.93E+04	13 %	2.96E+04	2.55E+04	14 %	6.08E+04	5.15E+04	15 %
*TRE*	*kg 1,4-DCB*	1.51E+05	1.43E+05	5 %	1.39E+05	1.34E+05	3 %	1.55E+05	1.45E+05	6 %
*HCT*	*kg 1,4-DCB*	1.43E+03	1.37E+03	4 %	1.15E+03	1.12E+03	3 %	1.23E+03	1160.17	6 %

Table 2 reveals a notable concentration of the total impact load in the HCT category. The remaining impact load is more equally distributed across the other impact categories.

#### 3.2.2 Midpoint level – characterisation

The characterization analysis was performed to compare each model with its respective optimized version. Through characterisation, potential hotspots were identified by assessing the contribution of each life cycle phase to the analysed impact categories. For each key phase identified, an analysis was conducted on the primary elementary flows that contribute to the overall burden of the specific impact category.

The article "Assessing the environmental performance of optimized commercial refrigerators with alternative refrigerants and remote monitoring system: A cradle-to-grave life cycle assessment" was published in 2024. Journal: Heliyon.

The results of the characterization of each selected impact category, obtained through normalisation for all models (standard and optimized), can be seen in Table 3.

The characterization reveals that the optimized versions demonstrated a significant reduction in environmental impacts across all impact categories. Notably, the FRS, FWE, and GWP exhibited the most substantial performance improvements.

The impacts of each lifecycle phase of the standard and optimized refrigerator versions are detailed in Table 4. The contributions are expressed in percentages of the total impact for each impact category. The percentage variation between the standard and optimized models is presented in the third column.

**Table 4:** Percentage characterization of life cycle phases for standard and optimized models and their variations. Cut-off contribution criteria of 1 %.

Model	Impact category	Standard in %			Optimized in %			Variation (Δ) in %	
		Raw Material	Transp	Use	Raw Material	Transp	Use	use	EoL
*A*	*GWP*	3 %	1 %	97 %	3 %	1 %	96 %	13 %	−148 %
	*FRS*	3 %	1 %	96 %	3 %	1 %	96 %	13 %	−57 %
	*FWE*	3 %	1 %	96 %	4 %	1 %	96 %	13 %	−49 %
	*TRE*	58 %	3 %	39 %	61 %	3 %	36 %	13 %	−41 %
	*HCT*	69 %	0 %	31 %	72 %	0 %	28 %	13 %	−84 %
*B*	*GWP*	10 %	1 %	88 %	12 %	1 %	86 %	16 %	−5%
	*FRS*	11 %	1 %	88 %	12 %	1 %	86 %	16 %	−6%
	*FWE*	15 %	1 %	84 %	17 %	1 %	81 %	16 %	−3%
	*TRE*	76 %	3 %	20 %	79 %	3 %	18 %	16 %	−6%
	*HCT*	81 %	0 %	18 %	84 %	0 %	16 %	16 %	−4%
*C*	*GWP*	4 %	0 %	95 %	4 %	0 %	95 %	16 %	16 %
	*FRS*	4 %	0 %	95 %	4 %	1 %	95 %	16 %	43 %
	*FWE*	5 %	0 %	94 %	6 %	0 %	93 %	16 %	22 %
	*TRE*	57 %	2 %	41 %	61 %	2 %	36 %	16 %	52 %
	*HCT*	62 %	0 %	38 %	66 %	0 %	34 %	16 %	55 %

The study revealed that materials had a substantial impact on two specific categories: TRE and HCT, as indicated in Table 4. Due to the complex nature of materials and processes in the raw materials phase, a detailed analysis was carried out specifically for these two impact categories, aiming to identify the main materials responsible for the impact load. The results are presented in Fig. 3.

**Fig. 3:** Characterization of the raw material phase for standard and optimized models.

The results presented in Fig. 3 represent the percentage contribution of materials from the raw material phase to the impact categories TE and HCT.

#### 3.2.3 Endpoint level

The ReCiPe Endpoint H/A method was calculated with the objective of obtaining a more comprehensive understanding of environmental effects, concentrating 18 impact categories into three distinct areas of concern: Human Health, Ecosystems, and Resources. The analysis results showed that, for all models, about 96 % of the impact burden of refrigerators is related to the Human Health protection area. Single score results are show in Table 5.

The article "Assessing the environmental performance of optimized commercial refrigerators with alternative refrigerants and remote monitoring system: A cradle-to-grave life cycle assessment" was published in 2024. Journal: Heliyon.

**Table 5:** Endpoint level single score results.

Models	Model A	Model A Optimized	Model B	Model B Optimized	Model C	Model C Optimized
Human Health	2.02	1.78	1.13	0.99	2.16	1.85
Ecosystems	1.93	1.71	1.08	0.95	2.07	1.77
Resources	0.07	0.06	0.04	0.03	0.07	0.06

## 4 Discussion

### 4.1 Refrigerator models

The results of the normalisation process, presented in Table 2, show that between 82 % and 87 % of the total burden in all models was concentrated in five impact categories: HCT, FRS, FWE, TRE, and GWP which were characterized.

The comprehensive life cycle analysis of all refrigeration systems clearly demonstrated that the Use Phase is the primary driver of impact across all impact categories, closely followed by the Raw Material Phase. The Use Phase, which corresponds to the operational period of the refrigerator, emerged as the major contributor due to the substantial energy consumption required for its operation, just as pointed out by other studies applied to the environmental analysis of refrigerators [13,42]. On the other hand, the Raw Material Phase encompasses the extraction and processing of the raw materials utilized in the production of the refrigerator.

The consumption of electricity during the use phase had a substantial impact on all identified impact categories, as indicated by the results presented in Table 4. Notably, the categories most affected were FRS, FWE, and GWP, which are directly linked to the production and distribution of electrical energy. These three categories collectively represented 81–97 % of the total impact load across all analysed models.

This highlights the substantial impact of current energy production in Europe. The European Power Grid relies on non-renewable primary energy sources, with 47 % coming from fossil sources and 38 % from nuclear power plants [43]. Specifically, electricity generation in Europe heavily relies on the utilization of lignite, natural gas, and hard coal, which have a substantial influence on FRS and GWP. It is worth noting that the use of lignite has the most pronounced impact on the FWE.

Specifically, European electricity generation relies heavily on the utilization of lignite, natural gas, and hard coal, which exert a substantial influence on FRS and GWP. Notably, the use of lignite has the most pronounced impact on the FWE category. Furthermore, the consumption of electricity contributed to a lesser extent, representing a total impact load of 16–41 %, to the categories of TRE and HCT. These impacts are primarily attributed to the infrastructure, materials used in construction (such as steel and copper), and the release of particulate matter resulting from the use of lignite and hard coal.

The article "Assessing the environmental performance of optimized commercial refrigerators with alternative refrigerants and remote monitoring system: A cradle-to-grave life cycle assessment" was published in 2024. Journal: Heliyon.

The extraction and processing of raw materials had a notable impact on the categories of TER and HCT, as demonstrated by Table 4. Specifically, the Raw Material Phase alone contributed to 57–84 % of the total impact load in these categories. Notably, Fig. 2 indicates that the use of two specific materials, steel, and copper, predominantly influenced these two categories, in accordance with reported by Rossi et al., 2021 [13]. HCT was primarily attributed to the use of steel, which is a major component in refrigerator manufacturing. The manufacturing process involving electric arc furnaces for steel production generates toxic slag, posing a significant risk to Human Health. On the other hand, TER is strongly associated with the use of copper in refrigerator heat exchangers, accounting for over 80 % of the impact in this category.

The other life cycle phases of all models had a minimal impact on the total impact load. Only the transportation phase showed an effect of 2–3% in the TRE category, mainly due to brake wear emissions. Upon analysing transportation separately, a significant association was observed with the HCT. In this case, the construction material of trucks, which is steel, along with fleet maintenance, diesel consumption, and road construction, emerged as the primary contributors to this impact category.

Based on the endpoint-level analysis, it was possible to corroborate the significant relative impact of the Use and Raw Material phases. The results clearly indicate that both phases predominantly contribute to the protection of Human Health. Approximately 96 % of the impact burden affects this area, which is directly associated with two of the primary impact categories identified as the most impactful through the normalisation process: GWP and HCT.

### 4.2 Comparison

Most of the inventory remained unchanged when comparing the standard and optimized models. The changes were primarily related to the replacement of the refrigerant and its end-of-life phase, as well as a negligible additional quantity of electronic components and sensors in Model C due to the installation of the WSMM system. The most significant change was observed in the consumption during the use phase. The optimization process with alternative refrigerants and the installation of the WSMM system resulted in substantial improvements in energy consumption reduction. By changing the refrigerant, it was possible to achieve an approximate 57 % reduction in energy consumption across all models. In Model C, with the installation of the WSMM system, it was possible to estimate the reduction in excess energy consumption caused by the compressor overload resulting from malfunction or damage to other components of the refrigeration system. In this case, an additional 3 % reduction was achieved due to the installation of WSMM equipment, representing a total consumption reduction of 60 % over the lifespan of Model C.

The article "Assessing the environmental performance of optimized commercial refrigerators with alternative refrigerants and remote monitoring system: A cradle-to-grave life cycle assessment" was published in 2024. Journal: Heliyon.

The study found that substituting R290 refrigerant with R744 in Model A resulted in an increase of up to eightfold in all impact categories, while Model B saw an overall increase of 18 %, and Model C experienced an overall reduction of 99 %. However, the overall impact load referent to the production, use, and refrigerant loss in the total impact was considered negligible as it represents less than 1 %. The main improvement was seen in the reduced electricity consumption during the use phase of optimized systems. The optimized models showed an average reduction in energy consumption of 57–60 % during the use phase, resulting in a reduction of approximately 13 % in Model A, 16 % in Model B, and around 16 % in Model C across all selected impact categories. Indeed, other LCA studies comparing the environmental performance of optimized refrigerator models with the substitution of more sustainable refrigerants have achieved significant improvements in the total impact load throughout the refrigerator's lifecycle. For instance, Rossi et al., 2021 [13] reported an improvement of approximately 10 % in environmental performance.

During the end-of-life phase, variations were observed in both standard and optimized models. Model A exhibited an increase in impact across all categories, ranging from 41 % to 147 %. This increase was attributed to the replacement of R290 refrigerant with R744. It is noteworthy that the standard Model A had 0.296 kg of propane as the refrigerant quantity. In contrast, the optimized Model A operated with a quantity of 1.5 kg of R744. A similar pattern was observed in Model B, where the only difference was an increase in the quantity of the same refrigerant, R744. In this case, the impact categories saw an approximate 5 % increase across the board. On the other hand, Model C, during its end-of-life phase, exhibited significant improvement with a reduction of 16 %–55 % in impact categories. Like Models A and B, this improvement stemmed from replacing R452A refrigerant with R290, resulting in a reduced quantity from 2.2 kg to 0.296 kg. However, it is important to emphasize that the observed improvements and drops in the different models are negligible, given that the contribution of the end-of-life phase to the overall impact load of refrigerators was less than 1 %. Similar findings have been reported in other studies [13,44], confirming the minimal impact of refrigerant usage compared to other phases in the lifecycle of refrigerators, especially the use phase.

The article "Assessing the environmental performance of optimized commercial refrigerators with alternative refrigerants and remote monitoring system: A cradle-to-grave life cycle assessment" was published in 2024. Journal: Heliyon.

During the end-of-life phase of a product's life cycle, recycling has proven beneficial for certain materials, as evidenced by studies conducted by Foelster et al., 2016 [45] and Xiao et al., 2016 [46]. These studies highlight the positive impact of recycling systems on refrigerators, particularly in terms of resource and energy savings for materials like polystyrene, steel, and copper. However, there are specific components, notably electronic ones, that contain substantial amounts of heavy metals and cannot be recycled [13,47]. For instance, electrical and electronic equipment can have significant consequences. Such equipment typically contains various toxic substances, including lead, mercury, cadmium, arsenic, selenium, chromium, cobalt, polychlorinated biphenyls, polyvinyl chloride, barium, beryllium, nickel, antimony, among others [48,49].

### 4.3 Sensitive analysis with alternatives functional unit

The sensitivity analysis for each analysed model regarding the alternative functional unit is presented in Table 6.

**Table 6:** Sensitive analysis comparing original and optimized scenarios.

Model		A			B			C		
Impact Category	Unit	Original (7 years)	Opt (10 years)	Variation	Original (7 years)	Opt (10 years)	Variation	Original (7 years)	Opt (10 years)	Variation
FRS	kg oil eq	1,07E+00	9,25E-01	14 %	3,49E-03	2,82E-03	19 %	4,06E-02	3,34E-02	17 %
FWE	kg P eq	4,55E-04	3,92E-04	14 %	1,32E-02	9,51E-03	28 %	8,98E-02	6,64E-02	19 %
GWP	kg CO2 eq	3,99E+00	3,44E+00	14 %	8,60E-07	7,04E-07	18 %	1,06E-05	8,78E-06	17 %
HCT	kg 1,4-DCB	1,29E-01	9,56E-02	26 %	7,32E-03	5,91E-03	19 %	8,48E-02	6,98E-02	18 %
TRE	kg 1,4-DCB	1,33E+01	1,00E+01	25 %	1,75E+00	1,44E+00	18 %	2,19E+01	1,81E+01	17 %

The results from Table 6 are expressed in terms of the alternative functional unit (liters refrigerated per year). When comparing the results of the alternative functional unit, a reduction in the impact load was observed in all analysed categories. Model A showed a decrease of 14–26 %, Model B exhibited a reduction ranging from 18 to 28 %, while Model C demonstrated a reduction of 17–19 %. This significant improvement in environmental performance can be attributed to the amortization of the most impactful life cycle phases (raw material and use phases) over 10 years, in addition to the optimization processes implemented in each of the models.

### 4.4 Limitations of the study

The LCA study was conducted using a combination of primary data and industry estimations, tailored to the availability of current databases. The model has been adjusted to adapt the limitations of the currently available databases (ecoinvent).

The article "Assessing the environmental performance of optimized commercial refrigerators with alternative refrigerants and remote monitoring system: A cradle-to-grave life cycle assessment" was published in 2024. Journal: Heliyon.

Parameters such as refrigerator energy consumption were calculated based on refrigerator power, without accounting for variations during real use. Furthermore, the impacts associated with component replacement were not considered. These aspects underscore the need for ongoing refinement and updates in LCA methodologies to ensure a more comprehensive and accurate assessment of environmental impacts.

## 5 Conclusions

The findings of this study highlight the importance of the Use and Raw Material Phase in refrigeration systems, as they emerged as the primary contributors to environmental impact across various impact categories. The Use Phase, driven by energy consumption, particularly electricity, was identified as the main source of impact. Fossil resource scarcity, Freshwater Eutrophication, and Global Warming were the most affected impact categories, with significant dependence on European energy production which is dependent on non-renewable primary energy fonts as fossil and nuclear sources. Furthermore, the extraction and production of raw materials, specifically steel and copper, played a crucial role in Terrestrial Ecotoxicity and Human Carcinogenic Toxicity.

The environmental benefits were primarily derived from energy savings achieved using alternative refrigerants, as well as the prevention of malfunctions and system damage facilitated by the installation of the WSMM system. These optimization strategies resulted in a significant reduction in electricity consumption during the Use Phase, positively impacting three key impact categories related to the production and distribution of electricity in the European grid: Fossil Resource Scarcity, Freshwater Eutrophication, and Global Warming.

Future research will certainly involve in-depth analyses of specific components within refrigeration systems, exploring optimization strategies, such as advanced technologies, materials, and operational practices, to ensure a more effective and sustainable approach in reducing the environmental footprint of refrigerators throughout their life cycle.

## Funding

This research was partially supported by ISA Spa (research contract with CIRIAF dated July 2nd, 2019, the results of which may be used by CIRIAF for scientific dissemination in journals).

## Data availability

The data pertinent to this investigation were not archived in a publicly repository. However, they can be accessed via the referenced sources and the ecoinvent V3.8 database. Additional data will be made available on request.

The article "Assessing the environmental performance of optimized commercial refrigerators with alternative refrigerants and remote monitoring system: A cradle-to-grave life cycle assessment" was published in 2024. Journal: Heliyon.

## CRediT authorship contribution statement

**Ramoon Barros Lovate Temporim:** Writing – review & editing, Writing – original draft, Methodology, Formal analysis, Data curation, Conceptualization. **Alessia Di Giuseppe:** Writing – review & editing, Visualization, Formal analysis, Data curation. **Fabiana Frota de Albuquerque Landi:** Writing – review & editing, Visualization, Methodology, Formal analysis, Data curation. **Andrea Nicolini:** Validation, Supervision, Resources, Project administration, Conceptualization.

## Declaration of competing interest

The authors declare that they have no known competing financial interests or personal relationships that could have appeared to influence the work reported in this paper.
